The article "Advertising Click-Through Rate Prediction Based on CNN-LSTM Neural Network" was retracted in 2023. Reasons: suspected computer-generated content; unreliable results or conclusions; concerns about the data; concerns about the results or conclusions.

# Advertising Click-Through Rate Prediction Based on CNN-LSTM Neural Network

**DOI:** 10.1155/2021/3484104

**Published:** 2021-08-13

**Authors:** Danqing Zhu

**Affiliations:** School of Arts & Communication, Xiamen Institute of Technology, Xiamen 361021, China

## Abstract

In the era of big data information, how to effectively predict and analyze the click-through rate of information advertising is the key for enterprises in various fields to seek returns. The point rate prediction of advertising is one of the core contents of advertising calculation. The traditional shallow prediction model cannot meet the nonlinear relationship of data processing, and the manual processing of data information extraction method is very resource consuming. To solve the above problems, this paper proposes a CNN-LSTM (convolutional neural network-long short-term memory) convolution hybrid neural network algorithm to predict the click-through rate of advertisements. According to the neural network algorithm, the prediction model is constructed, and the effective features are extracted in the process of model establishment, and the prediction analysis is carried out according to the simplified LSTM neural network time serialization features. CNN convolution neural network is used to train the prediction model. This paper analyzes the characteristics of traditional prediction methods and the corresponding solutions and carries out feature learning and prediction model construction for advertising click-through rate prediction. Then, the unknown behavior of advertising users is judged and predicted. The results show that, compared with the single structure network of traditional prediction model, the prediction effect based on CNN-LSTM neural network algorithm has higher accuracy.

## 1. Introduction

The development of online advertising began in the 1990s. This combination of network and information mainly changes the traditional way of information dissemination, from human propaganda to online advertising on the Internet, and the way of enterprise media's propaganda on their own industry has also changed [1]. The purpose of online advertising is to pay attention to every user and attract more users' attention through free use so as to achieve the promotion of industrial products and the dissemination of information [2]. Traditional advertising combined with the Internet can directly contact the characteristics and characteristics of users and become the core of information dissemination. Enterprises gain a lot of benefits through Internet advertising and soon find the differences between it and traditional media. It can analyze the characteristics of users, issue targeted ads, and push different types of targeted ads for different users [3]. This model greatly improves the efficiency of advertising. With the development trend of advertising, people gradually begin to pay attention to the click-through rate of advertising [4]. How to analyze people's interests and hobbies through the analysis of network big data to get people stop advertising information can be completed. Click-through rate refers to the ratio of the number of hits and the frequency of advertising. According to the effect and times of click-through rate of advertisement, enterprises decide the intensity and exposure time of such information publicity [5].

The article "Advertising Click-Through Rate Prediction Based on CNN-LSTM Neural Network" was retracted in 2023. Reasons: suspected computer-generated content; unreliable results or conclusions; concerns about the data; concerns about the results or conclusions.

At present, there are many research methods for advertising click-through rate prediction, such as predicting advertising click-through rate according to neural network algorithm and logical regression algorithm, and constructing quasi Newton training model [6]. This model is easy to analyze and explain the effect of the algorithm and usually acts on the basic standard of advanced model. SVM (support vector machine) model can process multilayer nonlinear data and distinguish them effectively [7]. However, SVM model cannot predict the accurate results of individual small base advertising data in big data. The dynamic network model is used to predict the click-through rate of advertising, and the model is established by combining the relevance of location information. Judge whether the click result occurs or not [8]. The FM model decomposition algorithm can also be used to learn the relationship between advertising features from different variables and classify the relationship. FM model is more intuitive than regression model [9]. In the future, the prediction method based on Lasso variable model can solve the problem of high difference and dispersion between information and data. The shallow learning feature is used to calculate the prediction data by statistical method to obtain the variable value of each layer and make the variables independent [10]. This way cannot express the relationship between internal relations. Then, based on the shallow traditional way, a neural network recursive algorithm is proposed. In the process of predicting the click-through rate, BP reverse algorithm is used to build the model [11]. The accuracy of this algorithm model is relatively high, but in the recursive descent process, there will be no problem in updating the variable parameters. Based on the above problems, we propose to use the time series function of LSTM neural network algorithm to predict the frequency of events [12].

LSTM long-term and short-term memory algorithm can provide accurate judgment basis for the prediction trend of time series [13]. At present, it has been widely used in various fields, such as advertising effect forecast, financial stock forecast, energy output forecast, and traffic data forecast. LSTM algorithm needs a large number of real-time data parameters in the prediction process, which increases the prediction process time [14]. For this kind of problem, many researchers put forward the method of simplifying the internal structure and produced a new standard LSTM simplified neural network structure. By using the joint input and forgetting curve simplification variant, the parameter variables and cost of the data model can be changed without reducing the performance of the algorithm. Then a control cycle unit gate based on reset and update function is proposed [15]. GRU control loop unit can achieve the same effect as LSTM model. And it has faster speed and higher efficiency in the analysis process of prediction results. Moreover, the model structure is simpler and uses fewer variables than the model structure of cyclic unit.

The article "Advertising Click-Through Rate Prediction Based on CNN-LSTM Neural Network" was retracted in 2023. Reasons: suspected computer-generated content; unreliable results or conclusions; concerns about the data; concerns about the results or conclusions.

At present, there are several problems in the process of advertising click-through rate prediction: first, we need to solve the problem of accuracy of prediction results. How to accurately evaluate the conversion efficiency of advertising is one of the important points of relative advertising [16]. However, due to the uncertainty and complexity of the audience, the results of advertising click will be affected by a variety of factors, such as how to determine the audience group of directional advertising, the display form and release time of advertising, etc. The second problem is the scattered distribution of big data [17]. In the face of massive data, how to select targeted and effective data samples for prediction and evaluation is also a problem we need to pay attention to [18]. In the loosely distributed data set, the advertising information that users interact with is very difficult to summarize; most of them are data without interaction traces. This situation leads to the advertising model being not able to directly contact with user interest. Finally, there is the problem of cooling transformation [19]. In the face of the situation that most new users and advertisements have no intersection, the accuracy of the prediction effect of the model will be affected. It directly leads to a sharp drop in the click-through rate of advertisements and the inability to track data information [20].

In this paper, we use CNN-LSTM convolution hybrid neural network algorithm to predict the click-through rate of advertisements and analyze the difference between traditional prediction model and deep learning neural network algorithm. This paper mainly uses the time series prediction method of LSTM neural network model and the simplified LSTM algorithm. This paper analyzes the prediction process and the structure of convolution hybrid neural network algorithm in the process of advertising click and studies the click rate prediction model. Finally, the experimental results of time series data set and CNN-LSTM neural network algorithm are analyzed.

The article "Advertising Click-Through Rate Prediction Based on CNN-LSTM Neural Network" was retracted in 2023. Reasons: suspected computer-generated content; unreliable results or conclusions; concerns about the data; concerns about the results or conclusions.

## 2. Research on Advertising Click-Through Rate Prediction Technology Based on CNN-LSTM Neural Network Algorithm

### 2.1. Research on CNN Convolutional Neural Network Technology and Time Series Technology of Simplified LSTM Neural Network

CNN is a neural network composed of multiple convolution layers and connection layers. The convolution unit of each level is neural unit [21]. Neural network algorithm is formed by convolution operation of neural unit. It can extract different parameter features. It is usually used in image processing, that is, to extract pixel information from the collected data graph. The disadvantage lies in the low-level features of intelligent data acquisition for input, such as edge, line, angle, etc. After multilayer network extraction and analysis, the final complex feature data can be obtained [22]. In the convolution weight matrix, feature points can be extracted in different ranges according to the same image feature [23]. The characteristic formula is as follows:

(1) $$\begin{array}{c} H_{i}=f\left(H_{i-1}⊗w_{i}+b_{i}\right), \end{array}$$

where *H*_*i*_ is the feature of the unknown layer, ⊗ is the convolution process operation, *w*_*i*_ is the weight variable of the unknown layer, and *b*_*i*_ is the offset position of the unknown layer. The convolution process of CNN is shown in Figure 1.

The white matrix in the figure represents the input information data. With the movement of the Yellow data on the white matrix, convolution is formed. Each time the convolution moves to a different position, the product of the generated element and its covered data will be corresponding. Finally, the integral results of the whole convolution matrix are accumulated into the pink matrix. The final convolution result is formed after all the motions pass a period.

According to the simplified standard LSTM network algorithm structure proposed by many scholars to reduce the degree of parameter redundancy, other models are proposed for comparison [24]. It is proved that the model can be transformed into LSTM model with less variables. By reducing the data of structural unit gate and updating unit gate, new variants are proposed, and the overall performance is analyzed. LSTM simplified neural network algorithm has the effect of time reduction and can use less comparative data for prediction and analysis [25].

The article "Advertising Click-Through Rate Prediction Based on CNN-LSTM Neural Network" was retracted in 2023. Reasons: suspected computer-generated content; unreliable results or conclusions; concerns about the data; concerns about the results or conclusions.

The basic LSTM neural network structure consists of three cell gates and one state element. The state element is used to store the object state data at that time. The structure unit gate is used to control the storage or discarding of data [26].

Formula (2) is the input signal calculation formula.

*x*_*t*_ is the real-time input data variable, *h*_*t*_ is the real-time output data variable, *Z*_*t*_ is the calculated input signal value, *w*_*z*_ is the weight in the input matrix, *U*_*z*_ is the weight in the recursive matrix, and *b*_*z*_ is the offset data value.

(2) $$\begin{array}{c} Z_{t}=g\left(W_{z}x_{t}+U_{z}h_{t-1}+b_{z}\right). \end{array}$$

Formula (3) is the calculation formula of input data:

(3) $$\begin{array}{c} i_{t}=\sigma \left(W_{i}x_{t}+U_{i}h_{t-1}+b_{i}\right). \end{array}$$

Equation (4) is the forgetting formula:

(4) $$\begin{array}{c} f_{t}=\sigma \left(W_{f}x_{t}+U_{f}h_{t-1}+b_{f}\right). \end{array}$$

Equation (5) is the state element formula:

(5) $$\begin{array}{c} c_{t}=f_{t}⊙c_{t-1}+i_{t}⊙z_{t}. \end{array}$$

Equation (6) is the output data formula:

(6) $$\begin{array}{c} o_{t}=\sigma \left(W_{o}x_{t}+U_{o}h_{t-1}+b_{o}\right). \end{array}$$

Equation (7) is the output signal calculation formula:

(7) $$\begin{array}{c} h_{t}=o_{t}⊙g\left(c_{t}\right). \end{array}$$

The variables in the above formula are the same as those in formula (2), which are the weight attributes in each matrix. Finally, the results of matrix variable point display are multiplied. On the premise of simplifying the structure of LSTM neural network model, this paper needs to analyze the standardized model. The internal structure of the standardized model is shown in Figure 2.

Based on the above formula, there are still three cell gates. Since the standard structure needs to calculate the variable dimension and the number of hidden units, the data will be superimposed every time the update operation is carried out. The simplified LSTM neural network model is modified according to the structure of joint input data element and forgetting unit. The data parameters involved in the calculation are simplified and updated to screen effective information. Remove redundant and duplicate data. Through this operation, the complex data sources faced by the neural network algorithm in the calculation process are reduced, so as to improve the speed of learning and training data [27]. In the process of controlling the input data element, it is necessary to input the obtained network information. This model is the same as the traditional standard structure network. The calculation formula is as follows:

(8) $$\begin{array}{c} z_{t}=\sigma \left(W_{z}x_{t}+U_{z}h_{t-1}+b_{z}\right),\\ i_{t}=\sigma \left(W_{i}x_{t}+U_{i}h_{t-1}+b_{i}\right). \end{array}$$

The state metadata is updated by comparing the input data with the last control legacy state element. The updated formula is as follows:

(9) $$\begin{array}{c} c_{t}=\left(1-i_{t}\right)⊙c_{t-1}+z_{t}. \end{array}$$

It can be seen that the simplified version of neural network has different characteristics from the standard version. Instead of forgetting unit, the above formula can selectively store the state data. When the value is 0, all the state data of the previous time are recorded. When the value is 1, forget all the state data of the previous time. In this way, the input state and forget state are fused. When the data is input and removed, the data is output. The state element controls the data output of the previous time, and the structure is the same as that of the standard neural network. The formula is as follows:

(10) $$\begin{array}{c} o_{t}=\sigma \left(W_{o}x_{t}+U_{o}h_{t-1}+b_{o}\right),\\ h_{t}=o_{t}⊙g\left(c_{t}\right). \end{array}$$

It can be seen that the output unit controls the data output of LSTM neural network algorithm at the last moment. If the data value *o*_*t*_ is 0, the last time state element cannot be output, and the value of *h*_*t*_ is 0. If *o*_*t*_ data value is 1, all the last time state metadata will be displayed. After the combination of input data and forgetting unit, LSTM neural network is transformed from standardized structure to simplified structure, and then from three-unit gate structure to two-unit gate structure. Each time the data stack process needs to change, more variable parameters also change. Compared with the standard structure, the calculated value is reduced by a quarter. Although the combined input data unit gate and forgetting unit gate simplify the operation of the standard LSTM neural network, in each learning process, we need to update the matrix data again. This kind of processing will lead to the increase of the calculation value and consume a long time. On the basis of no loss of efficiency and accuracy, we further propose a method to reduce the learning time. The first is to simplify the I-type neural network, in addition to deleting the weight value of input and output data to simplify the process. The matrix formula is as follows:

(11) $$\begin{array}{c} \left\{\begin{array}{c} z_{t}=g\left(W_{z}x_{t}+U_{z}h_{t-1}+b_{z}\right),\\ i_{t}=\sigma \left(U_{i}h_{t-1}+b_{i}\right),\\ c_{t}=\left(1-i_{t}\right)⊙c_{t-1}+z_{t},\\ o_{t}=\sigma \left(U_{o}h_{t-1}+b_{o}\right),\\ h_{t}=o_{t}⊙g\left(c_{t}\right). \end{array}\right. \end{array}$$

As can be seen from formula (11), the difference between the simplified I-type neural network structure and the standard version is that the data processing of the control gate is controlled by the time signal. The parameter values of the weight matrix and the offset matrix need to be updated in the process of hierarchical superposition decrease, which reduces the difficulty of the overall calculation. The internal diagram of the simplified version of LSTM neural network is shown in Figure 3.

The article "Advertising Click-Through Rate Prediction Based on CNN-LSTM Neural Network" was retracted in 2023. Reasons: suspected computer-generated content; unreliable results or conclusions; concerns about the data; concerns about the results or conclusions.

### 2.2. Research on CNN-LSTM Convolutional Neural Network Adding Attention Mechanism Model for Prediction

Firstly, the advertising prediction model is evaluated exponentially, and the click-through rate prediction model is an interactive activity process. We use the evaluation index in the field of training and learning, that is, accuracy and recall rate. In order to deal with the model factors in the comprehensive factor environment, the accuracy curve and characteristic curve are used to evaluate the model ability in the research process. Based on the use of attention mechanism model in deep learning neural network algorithm, we combine dynamic network with users' click interest in advertising. Build a dynamic click-through rate prediction model with the change of user interest. The model can comprehensively calculate the user's interest characteristics when selecting ads according to the user's footprint information and historical browsing. The obtained information data is defined as variables and added to the calculation process of attention mechanism. Attention mechanism in the field of neural machine as a translation function has achieved good feedback, through the control matrix parameters according to user footprints and relationship analysis to calculate the next run. Din model is the use of attention mechanism to improve the performance of data information construction model and click-through rate prediction. This model analysis shows that there is a correlation between the user's footprint behavior and the characteristics of clicking on ads or viewing news at the latest time. According to the user's interest, the corresponding measures can improve the number of clicks. Din structure uses attention mechanism to improve the internal structure layer, and the changed structure produces differentiated variable output according to the user's interest characteristics. It enhances the display ability of the construction model after the analysis of user characteristics. However, the defect of DIN model is that it cannot analyze the dynamic and time-varying characteristics of users' concerns.

Based on deep learning neural network and attention mechanism DIN model, we combine the dynamic characteristics of users with click-through rate prediction to form a new DIPN model. According to the user's footprint characteristics, DIPN calculates the number of hits and the characteristics of the viewed ads and predicts the user's advertising interest points. The data results are combined with the weight variables of attention mechanism to calculate. Then the DIPN model is combined with CRU layer to improve the efficiency of recording feature points. The structure diagram of DIPN model is shown in Figure 4.

The article "Advertising Click-Through Rate Prediction Based on CNN-LSTM Neural Network" was retracted in 2023. Reasons: suspected computer-generated content; unreliable results or conclusions; concerns about the data; concerns about the results or conclusions.

In the model, the input of footprint query can display the advertising information that users have browsed including viewed and not viewed advertising information. DIPN uses deep learning algorithm to calculate interest curve according to historical data, as shown in Figure 5.

Among them, the positive curve represents the advertising news that users like and are interested in, and the negative curve represents the advertising news that users do not browse or view. According to the interest curve, the click data is extracted from the footprint features and added to the calculation vector. Firstly, the GRU layer model is used to display the interest features in the footprint information, and then the hidden state computation and the predicted advertising vector are used as the calculation variables of the attention mechanism layer. The formula of d-softmax function is as follows:

(12) $$\begin{array}{c} a_{ij}=\frac{e^{dx_{i}}}{\sum_{i=1}^{n}e^{dx_{i}}}. \end{array}$$

The data object represents the degree of user's interest in advertising in the algorithm and contains each element of the characteristic variable when the attention mechanism outputs the network layer.

Before studying the process of advertising click-through rate prediction, this paper first analyzes the overall framework. The prediction process includes raising problems, storing data sources, solving problems, estimating click-through rate, feature learning, model building, index acquisition, and other processes. The advertising click-through rate prediction framework is shown in Figure 6.

The existing problems are sparse distribution of data sources. We can analyze the data by decomposing the matrix to calculate the vector. Or machine learning algorithm is used to deal with the data sparsity problem according to the decomposition degree of the model and the interaction between vector and feature. Aiming at the problem of uneven data sources, the problem is solved from the source. In the process of collecting and storing information, the source data is sampled by distribution, so that the difference of the whole data will not be too big. Firstly, the positive vector samples are collected, and then the negative vector samples are collected. The data obtained are converted into input model data after training. This average data source method can reduce the repeatability and unconsciousness of vector samples, reduce the training time, and improve the overall prediction speed. Based on CNN-LSTM convolution hybrid neural network algorithm, the process of advertising click-through rate prediction becomes much simpler. The main steps are as follows: firstly, feature analysis and extraction are carried out on the data source, and the feature points that have an impact on the click-through rate are obtained by using the interest processing method, and then the cutting training is carried out. Secondly, the vector model is constructed to input the training data, and the simplified algorithm is used to calculate the model data. Finally, the simplified data set of the model is input into the prediction algorithm to get the result feedback given by the prediction system, and the ranking result is used to determine the position and direction of the news advertisement. The simplified process is shown in Figure 7.

The article "Advertising Click-Through Rate Prediction Based on CNN-LSTM Neural Network" was retracted in 2023. Reasons: suspected computer-generated content; unreliable results or conclusions; concerns about the data; concerns about the results or conclusions.

First of all, regression algorithm can be used to classify classical models, which can solve linear or nonlinear classification problems and can be divided into multiple categories. Among them, the formula of decision-making function can be in many forms:

(13) $$\begin{array}{c} \varpi^{T}x+b=\sum_{i=1}^{n}\varpi_{1}x_{1}+\cdots +\varpi_{n}x_{n}+b. \end{array}$$

By expanding the calculation and adding the square root of the variable, we can know the nonlinear calculation formula in the logistic regression algorithm:

(14) $$\begin{array}{c} \varpi_{1}x_{1}+\varpi_{2}x_{1}^{2}+\cdots +\varpi_{2n-1}x_{n}+\varpi_{2n}x_{n}^{2}+b, \end{array}$$

*ϖ* is the weight variable, *x* is the input data, and *b* is the offset data. In the process of advertising click, whether there is click operation is a problem of ambiguity, which has the nature of classification. When the probability of *Y*=1 is the hit rate, the ambiguity property can be expressed as the parameter *μ* by binomial distribution:

(15) $$\begin{array}{c} p\left(h\right)=\mu^{h}{\left(1-\mu \right)}^{1-h}. \end{array}$$

The advertising click-through rate prediction model can establish a functional relationship between the feature points and the click-through parameter *μ*. The probability model is as follows:

(16) $$\begin{array}{c} p\left(Y=1|x\right)=\frac{\exp\left(\varpi^{T}x+b\right)}{1+\exp\left(\varpi^{T}x+b\right)},\\ p\left(Y=0|x\right)=\frac{1}{1+\exp\left(\varpi^{T}x+b\right)}. \end{array}$$

A variable value of 1 represents a positive vector sample, and a variable value of 0 represents a negative vector sample. For the training process of multicombination data, the maximum likelihood parameter can be estimated, and the maximum function is as follows:

(17) $$\begin{array}{c} L\left(\varpi \right)=\sum_{i}^{N}\left[y_{i}\left(\varpi^{T}x_{i}\right)-\mathrm{lg}\left(1+\exp\left(\varpi^{T}x_{i}\right)\right)\right]. \end{array}$$

The maximum likelihood function is used as the calculation formula to get the optimal data form. *L*(*ϖ*) is the maximum and *ϖ* is the predicted value.

The article "Advertising Click-Through Rate Prediction Based on CNN-LSTM Neural Network" was retracted in 2023. Reasons: suspected computer-generated content; unreliable results or conclusions; concerns about the data; concerns about the results or conclusions.

Based on CNN-LSTM convolution hybrid neural network model, the hit rate prediction structure is divided into three layers. The first layer is deduplication and deburden coding, according to the encoded vector data to obtain new feature points. In the second layer, the feature points are input into the network model, and convolution and pooling layers are set. Through convolution distribution and weight variable analysis, the relationship between feature points is obtained. In the third layer, the convolution output is used as the input value of the simplified LSTM algorithm. Finally, the prediction value of the click-through rate of the advertisement is obtained by using the classification cutting function. The process is shown in Figure 8.

## 3. Analysis of Research Results Based on CNN-LSTM Neural Network Algorithm

### 3.1. Analysis of Time Series Prediction Results of Simplified LSTM Neural Network Algorithm

We need to verify the time series prediction results of the simplified neural network algorithm structure. The RMSE prediction model is used to study the accuracy. The formula is as follows:

(18) $$\begin{array}{c} \text{RMSE}=\sqrt{\frac{\sum_{t=1}^{N}{\left(h_{d,t}-h_{t}\right)}^{2}}{N}}. \end{array}$$

The sample data of the formula are rational numbers, and the ability of this model is compared with many models, such as the standardized neural network algorithm, the simplified structure algorithm of cell gate, the network structure algorithm of only removing the weight matrix, and so on. Firstly, the training calculation and result test are carried out under the condition that the variable parameters are consistent with the learning efficiency, dimensions, training data, and other objects. The experimental process was carried out more than 20 times, and the average of the results was taken. Two time series basic data combinations are set to predict the performance. In this study, all the sample data generated are predicted by time series. The first 2000 parts are training control group, and the last 3000 parts are experimental control group. The RMSE curve of LSTM simplified training process is shown in Figure 9. The test results are shown in Figure 10.

The article "Advertising Click-Through Rate Prediction Based on CNN-LSTM Neural Network" was retracted in 2023. Reasons: suspected computer-generated content; unreliable results or conclusions; concerns about the data; concerns about the results or conclusions.

According to the experimental results, it can be seen that the simplified LSTM neural network algorithm can quickly get all the prediction data. The fitting effect can also get the average distribution. The performance comparison of different models is shown in Table 1.

It can be seen from Table 1 that the simplified structural model can shorten the prediction time by reducing the parameter data, and the time of using the simplified I-type data which needs to be updated is obviously shorter than that in the case of large number of variants. The results show that the simplified structure model can make LSTM neural network algorithm shorten the prediction time and reduce the complexity of the calculation process while ensuring the accuracy.

### 3.2. Experimental Results Analysis of Convolution Hybrid Neural Network Algorithm Based on CNN-LSTM

Firstly, the data source is introduced. The data source used in the experiment is open source data. The data dimension is uniform degree. It includes continuous feature points and special feature points. The variable values are positive and negative samples, and the proportion of positive samples in the initial data source is similar, which will not affect the results. Secondly, the curve of the feature is analyzed according to the AUC index, and the ROC curve is calculated by the limit of the threshold. With the increase of the number of variables and the number of layers of the feature map, the more obvious the feature points are, the more complex the process of neural network algorithm is. In this case, the consumption of training time will also increase. In the comparison between CNN-LSTM neural network algorithm and other algorithms, four algorithms are selected for comparison. They are Adam algorithm, momentum algorithm, Adagrad algorithm, and SGD algorithm. Therefore, we need to choose the appropriate variable parameters for calculation. When selecting the optimal data variables, the experiment found that the number of LSTM layers, the training effect of the model, the optimal method, and the output dimension had a significant impact on the experimental results [28]. The results are shown in Figure 11. The experimental environment configuration is shown in Figure 12.

In this experiment, the deep and shallow models are used to predict the click-through rate of advertisements, and the results show that the deep model is better than the traditional model. The prediction system based on convolution hybrid neural network algorithm has better performance than single CNN algorithm or standard LSTM algorithm. The time consumed in the training process is also more than that of a single structure.

The article "Advertising Click-Through Rate Prediction Based on CNN-LSTM Neural Network" was retracted in 2023. Reasons: suspected computer-generated content; unreliable results or conclusions; concerns about the data; concerns about the results or conclusions.

## 4. Conclusion

With the development of Internet technology, in order to meet people's needs and interests, enterprises will carry out targeted advertising when carrying out advertising. In this paper, based on CNN-LSTM neural network algorithm to predict the click rate of advertising experimental research and analysis, firstly, the prediction and transformation process of click-through rate are introduced, and the algorithm structure of CNN convolution neural network is analyzed. Secondly, the results of the standard LSTM neural network algorithm and the simplified algorithm are compared, and it is concluded that the simplified neural network model has faster efficiency and lower consumption in the prediction and analysis process. By capturing the data source to study the sparsity problem, it can be found that the click rate prediction problem is changing in a variety of feature network structures. Finally, in the experimental analysis of convolution hybrid network algorithm, it is found that the prediction effect of this model is significantly higher than that of the traditional prediction model. The feature points extracted by convolution motion and hybrid algorithm can reduce manpower and time consumption. It can effectively improve the accuracy and efficiency of advertising prediction [29].

## Figures and Tables

**Figure 1:** CNN convolution operation process chart.

**Figure 2:** Internal structure diagram of standardized model.

**Figure 3:** Internal structure diagram of LSTM neural network.

**Figure 4:** DIPN model structure diagram.

**Figure 5:** Interest curve.

**Figure 6:** Advertising click-through rate prediction framework.

**Figure 7:** Simplified advertising forecast flow chart.

**Figure 8:** Algorithm structure diagram of convolution hybrid neural network.

**Figure 9:** RMSE curve.

**Figure 10:** Test result chart.

**Figure 11:** Comparison of parameters.

**Figure 12:** Experimental environment configuration.

**Table 1:** Performance comparison of different models.

Model	RMSE		Training time	Number of parameters
	Training sample	Test sample		
Standard LSTM	0.0600	0.0793	98.67	384
Variant I	0.0600	0.0741	73.91	288
Variant II	0.0600	0.0733	72.68	192
Variant III	0.0600	0.0708	92.62	128
Simplified I	0.0600	0.0752	58.68	144
Simplified II	0.0660	0.0781	69.05	96

## Data Availability

All the data of this study are from the big data statistics of the test process. The data of this paper can fully support the research results of this paper.
